The article "Stability Study and Simulation of Quadruped Robots with Variable Parameters" was published in 2022. Journal: Appl Bionics Biomech.

# Stability Study and Simulation of Quadruped Robots with Variable Parameters

**DOI:** 10.1155/2022/9968042

**Published:** 2022-01-19

**Authors:** Qian Cong, Xiaojie Shi, Ju Wang, Yu Xiong, Bo Su, Wei Xu, Hai Liu, Kuiyue Zhou, Lei Jiang, Weijun Tian

**Affiliations:** ^1^Key Laboratory of Bionic Engineering, Ministry of Education, Jilin University, Changchun 130022, China; ^2^China North Vehicle Research Institute, Fengtai District, Beijing 100072, China; ^3^College of Biological and Agricultural Engineering, Jilin University, Changchun 130022, China

## Abstract

Walking stability is one of the key problems restricting the development of quadruped robots. Two new kinds of variable parameter quadruped robots with high stability were proposed. The two groups of variable parameter models were applied to quadruped robots with the full elbow joint or elbow joint for front legs and knee joint for back legs, respectively, and the stability of their linear motion under different variable parameters was deeply studied by Recurdyn. The quadruped robots with elbow joint for front legs and knee joint for back legs displayed good antijamming ability to lateral impact. According to the rigid-flexible simulation experiment, the largest force occurred in the knee joint during the movement of the quadruped robot. This provided a theoretical basis for the design of real quadruped robots.

## 1. Introduction

As evolved and diverse creatures on land, quadrupeds have many advantages such as high power, adaptability, stability, and load capacity and can reach almost any region on the earth's land [1–5]. Inspired by quadrupeds, a variety of quadruped robots have been designed and built to play a role in a wide range of fields, including military reconnaissance, resource exploration, and disaster relief [6–10]. The study of kinematics and dynamics of quadruped robots has been a hot spot since they were born [11–13], especially in walking stability [2, 14, 15]. Payandeh et al. examined the influence of planning parameters on quadruped robots' stability. They found that it would improve the stability by adding lateral and longitudinal motion [16]. Sabelhaus et al. reported a kind of walking quadruped robot with the spine to enhance stability, which could lift the foot to over obstacles by bending and rotation movements [17]. Han et al. camp up with a trot gait planning method for quadruped robots, which improved walking stability by changing the optimal initial position of the supporting foot [18]. Chen et al. proposed a compliant control method for hydraulic actuated quadruped robot. The experimental results showed that this method can help the robots not only walk stably and climb hills but also resist a certain lateral impact [19]. In order to improve the flexibility and stability of movement, Zhang et al. proposed a quadruped robot with a moveable trunk. The robot could twist the trunk like a quadruped animal and obtained good stability margin [20].

Although the walking stability of quadruped robots achieved good results [21, 22], there are still some problems waiting to be solved. Lots of researches focused on the movement law and movement force of the legs by fixing the robot body. Thus, the interaction between the leg structures and the body in the whole movement could not be fully considered in the real movement [23]. Some studies focused on the static stability, the stability margin, and so on, but the simulation results were not very satisfactory [24]. Aiming at the deficiencies of these studies, two variable parameter quadruped robots are established and their walking stability is tested. Most quadruped animals have the compound characteristics of the full elbow joint or elbow joint for front legs and knee joint for back legs [25, 26]. The walking performances of quadruped robot with full elbow joint and elbow joint for front legs and knee joint for back legs are better than that of full-knee and external knee-elbow robots, and most quadruped robots adopt the first two designs [5, 27–29]. Therefore, the quadruped robots with the above two leg configurations are selected as our research objects. The dynamic rigid-flexible coupling simulation is used to analyze the force on the legs of the quadruped robot with variable parameters during the whole movement. Finally, the optimal configuration of quadruped legs under different movement conditions is obtained.

## 2. Design of Quadruped Robots with Variable Parameters

The motion of the thigh and calf in quadruped robots was displayed in Figure 1. In the whole swing phase, the thigh and calf would swing at the same time. The equivalent motion method was used to analyze the composite movement of thigh and leg by stages. The swing angle of the thigh was *A*_1_, the swing angle of the calf was *A*_2_, and the speed was *v*. *S* was stride length, and *T* was walking period. The length of thighs and calves were *L*_1_ and *L*_2_, respectively. The initial position of hip and knee joints were *θ*_1_ and *θ*_2_. *θ*_1_ = 60°, and *θ*_2_ = 30°. According to the geometric relationship [30], the following formulas can be obtained:

(1) $$\begin{array}{c} \left\{\begin{array}{c} L=L_{1}\cos\theta_{1}+L_{2}\cos\theta_{2},\\ S=\frac{Tv}{2},\\ \sin A_{1}=\frac{\text{S}}{2L}, \end{array}\right. \end{array}$$

(2) $$\begin{array}{c} \cos\left(\theta_{2}+A_{2}\right)=\frac{\left(L_{2}*\cos\theta_{2}-h\right)}{L_{2}}. \end{array}$$

Quadruped robots should have enough distances between their feet and the ground to prevent contacting interference. The foot clearance was set a maximal height *h* = 0.02 m at the midpoint of swing phase, got from Figure 1. The design parameters of this model were as follows: *L*_1_ = 0.2 m and $L_{2}=0.2\sqrt{3}$ m. *v* was mainly determined by *A*_1_, while the obstacle crossing ability of the quadruped robot (*h*_max_) was mainly determined by *A*_2_.

Walking speed and period were set as independent variables in simulation design. When *T* = 1 s, *v* was set as 0.1 m/s, 0.3 m/s, 0.5 m/s, and 0.7 m/s, respectively. When *v* = 0.3 m/s, *T* was set as 0.2 s, 0.4 s, 0.6 s, and 0.8 s, respectively. The simulation results are shown in Tables 1 and 2. It could be seen from Tables 1 and 2 that the contribution rate of *A*_2_ to *v* was 0%, and that of *A*_1_ to *v* was 100%.

For smoothness of walking, the hip joint was driven by sine function and the knee joint was driven by half wave function [31]. In the motion gait of quadrupeds, tort gait had been proved to have not only strong motion stability but also low energy expenditure. Therefore, tort gait was used in the proposed quadruped robots. The motion of diagonal hip joints in quadruped robots was the same, and their phase difference was *T*/2. In the beginning, the front and back hip joints in one side should be in the maximum phase in opposite directions. The model of quadruped robots with elbow joint for front legs and knee joint for back legs was taken as an example. The joint driving function is shown in Equations (3) and (4).

(3) $$\begin{array}{c} F_{1}\left(x\right)=A_{1}*2*\frac{pi}{360}*\sin\left(2*\frac{pi}{T}*x+\frac{\pi }{2}\right), \end{array}$$

(4) $$\begin{array}{c} F_{2}\left(x\right)=A_{1}*2*\frac{pi}{360}*\sin\left(2*\frac{pi}{T}*x-\frac{\pi }{2}\right). \end{array}$$

The function value of driving functions for knee joints facing forward should be positive while that of knee joints facing backward should be negative. The knee joint driving function is shown in Equations (5) and (8).

(5) $$\begin{array}{c} F_{3}\left(x\right)=A_{2}*2*\frac{pi}{360}*\frac{\sin\left(2*pi/T*x\right)}{2}+\left|\left.A_{2}*2*\frac{pi}{360}\frac{\sin\left(2*pi/T*x\right)}{2}\right|,\right. \end{array}$$

(6) $$\begin{array}{c} F_{4}\left(x\right)=A_{2}*2*\frac{pi}{360}*\frac{\sin\left(2*pi/T*x+pi\right)}{2}+\left|\left.A_{2}*2*\frac{pi}{360}*\frac{\sin\left(2*pi/T*x+pi\right)}{2}\right|\right., \end{array}$$

(7) $$\begin{array}{c} F_{5}\left(x\right)=-A_{2}*2*\frac{pi}{360}*\frac{\sin\left(2*pi/T*x+pi\right)}{2}-\left|\left.A_{2}*2*\frac{pi}{360}*\frac{\sin\left(2*pi/T*x+pi\right)}{2}\right|\right., \end{array}$$

(8) $$\begin{array}{c} F_{6}\left(X\right)=-A_{2}*2*\frac{pi}{360}*\frac{\sin\left(2*pi/T*X\right)}{2}-\left|\left.A_{2}*2*\frac{pi}{360}*\frac{\sin\left(2*pi/T*X\right)}{2}\right|.\right. \end{array}$$

*A*_1_, *A*_2_, and *T* in the above functions were taken as values listed in Tables 1 and 2, respectively, for the simulation experiment. The knee joint driving functions of quadruped robots with full elbow joint are shown in Equations (5) and (6).

Quadruped robots were built in CATIA, and the interference detection was carried out. The length of quadruped robots' leg and thigh was set to 200 mm and 350 mm. The foot end was a half-sphere with a diameter of 20 mm. The friction coefficient in the simulations was determined according to the contact materials. From Figure 2, the motion curve was quite smooth and periodic, indicating that proposed quadruped model could walk stably.

## 3. Results and Discussions

As shown in Figures 3 and 4, when *T* = 1 s, *v* was high, and the straight walking stability of quadruped robots with front legs and knee joint for back legs would be reduced. When *v* = 0.3 m/s, they had the best straight walking stability and the lowest lateral slip rate *U*. *U* was defined as shown in Equation (9). *S*_*x*_ was the real longitudinal distance of the quadruped robot while *S*_*y*_ was the lateral one. When *v* = 0.5 m/s, *U* = 30%, resulting in severe lateral slip. When quadruped robots with front legs and knee joint for back legs walked at constant period *T*, there was no linear relationship between the stability of straight walking and *v*, but there was an optimal value of speed to get the best stability. There was a similar relationship between walking efficiency *W* and *v*, and the optimal speed was 0.3 m/s. *W* was defined as shown in Equation (10). *S*_*T*_ was the theoretical longitudinal distance of quadruped robots.

(9) $$\begin{array}{c} U=\frac{S_{y}}{S_{x}}\times 100\%, \end{array}$$

(10) $$\begin{array}{c} W=\frac{S_{x}}{S_{T}}\times 100\%. \end{array}$$

As shown in Figures 5 and 6, when quadruped robots with front legs and knee joint for back legs walked at constant speed *v*, there was no linear relationship between the stability of straight walking and *T*, but there was an optimal value of period to get the best stability. When *T* was 0.2 s, *U* was smaller, and quadruped robots had a very good ability to walk. The relationship between the longitudinal walking distance and period is displayed in Figure 6 (*v* = 0.3 m/s). When *T* = 0.4 s, the longitudinal distances of quadruped robots with elbow joint for front legs and knee joint for back legs were large. After that, the longitudinal displacement did not increase, even if the period was longer.

The simulation results of full-elbow quadruped robots are displayed in Figures 7–10. When *T* = 1 s and *v* = 0.1 m/s, *U* had a minimum value of about 0.8%. When *v* = 0.7 m/s, although the longitudinal distance was largest, the lateral slip rate was largest, which indicated robots with full elbow joint would have severe slippage during the walking process and no longer maintain a stable walking state. When the period was constant, there was an optimal speed to make full-elbow quadruped robots walk stably.

The lateral slip rate of full-elbow quadruped robots increased with the walking period when *v* = 0.3 m/s. Through the comparison, it can be clearly concluded that under the condition of given walking speed, the full-elbow quadruped robot had better walking stability under the condition of relatively small walking period.

In the real environment, uneven ground, obstacles and external impacts brought many difficulties to real applications of quadruped robots. The impact resistance test was conducted under the condition of *T* = 1 s and *v* = 0.1 m/s. The mass of the robot was 320 kg. The impact (600 N) was applied in the barycenter of robots when the left front foot and the right hind foot were in the supporting phase, and the right front foot and the left hind foot were in the swinging phase. The impact force was applied to the left side of the robot instantaneously.

It could be seen from Figures 11 and 12 that when quadruped robots with full elbow joint received lateral impact force, the fuselage turned over. However, when subjected to the same impact force, quadruped robots with elbow joint for front legs and knee joint for back legs only experienced a short lateral deviation and then kept their original walking pattern and continued to walk steadily.

As shown in Figure 13(a), when the lateral force was applied to the barycenter of robots' fuselage, there was a distance between fuselage barycenter and the barycenter of quadruped robots with full elbow joint in the horizontal direction, so the torque (*T*) generated by the impact on the barycenter can be divided into *T*_*x*_ and *T*_*y*_. As shown in Figure 13(b), the barycenter of quadruped robots with full elbow joint and that of the fuselage were in the same straight line in the vertical direction, so *T* = *Ty*. When the barycenter of the body was subjected to lateral force, quadruped robots with elbow joint would be subjected to one more torque *T*_*x*_ than the other quadruped robots, so their impact resistance ability was weaker. It was clearly seen from Figure 14 that the walking distance of quadruped robots with full elbow joint was greater than that of quadruped robots with elbow joint for front legs and knee joint for back legs, indicating that quadruped robots with elbow joint for front legs and knee joint for back legs had serious slipping phenomenon when walking in a straight line.

The rigid-flexible coupling models of quadruped robots were established in Recurdyn to analyze their stress state. The stress on the four legs of the quadruped robot was similar in the motion, so only the force on the right front leg was analyzed to improve the speed of simulation calculation. The simulation results displayed that the maximum force in the quadruped robot occurred when the legs change from swing phase to support phase. Specifically, the stress was maximum when the leg began to fall to the foot and contact with the ground. The stress on the robot was concentrated near the knee joint, and the stress on the thigh was greater than that on the calf (Figure 15). The maximum pressure of the full-elbow quadruped robot (17.42 MPa) was much smaller than of quadruped robots' elbow joint for front legs and knee joint for back legs (36.51 MPa).

## 4. Conclusions

Two novel quadruped robots with variable parameters were presented. The joint driving functions of quadruped robots were proposed which were based on the kinematics model of quadruped robots. The walking stability and motion of quadruped robots with full elbow joint and elbow joint for front legs and knee joint for back legs were studied by simulations. The walking stability of full-elbow quadruped robots was better than that of the other when they were subjected to the same lateral impact on the barycenter of bodies. The main stress parts of proposed quadruped robots were the thigh parts. The stress on the thigh in quadruped robots with full elbow joint was less than that of quadruped robots with elbow joint for front legs and knee joint for back legs. All in all, these two kinds of quadruped robots have their own unique advantages, suitable for different application environment. This research provides a solid theoretical basis for the manufacture and development of quadruped robots with high stability in the future.

## Figures and Tables

**Figure 1:** Motion of robots.

**Figure 2:** Foot motion track of quadruped robot with (a) elbow joint for front legs and knee joint for back legs and (b) full elbow joint.

**Figure 3:** Lateral distance of quadruped robots with elbow joint for front legs and knee joint for back legs with different speed at a constant period.

**Figure 4:** Longitudinal distances of quadruped robots with elbow joint for front legs and knee joint for back legs with different speed at a constant period.

**Figure 5:** Lateral distances of quadruped robots with elbow joint for front legs and knee joint for back legs with different period at a constant speed.

**Figure 6:** Longitudinal distances of quadruped robots with elbow joint for front legs and knee joint for back legs with different period at a constant speed.

**Figure 7:** Lateral distances of quadruped robots with full elbow joint with different speed at a constant period.

**Figure 8:** Longitudinal distances of quadruped robots with full elbow joint with different speed at a constant period.

**Figure 9:** Lateral distances of quadruped robots with full elbow joint with different period at a constant speed.

**Figure 10:** Longitudinal distances of quadruped robots with full elbow joint with different period at a constant speed.

**Figure 11:** Movement of quadruped robots with full elbow joint under lateral impact.

**Figure 12:** Movement of quadruped robots with elbow joint for front legs and knee joint for back legs under lateral impact.

**Figure 13:** Schematic diagram of torque analysis in quadruped robots with (a) full elbow joint and (b) elbow joint for front legs and knee joint for back legs.

**Figure 14:** Motion distance of the center of mass of (a) full elbow joint and (b) elbow joint for front legs and knee joint for back legs under the interference of lateral impact.

**Figure 15:** Rigid-flexible coupling dynamic simulation results.

**Table 1:** Simulation results of walking with fixed period.

*v* (m/s)	0.1	0.3	0.5	0.7
*A*_1_	3.6°	10.8°	18.2°	25.9°
*A*_2_	6.1°	6.1°	6.1°	6.1°

**Table 2:** Simulation results of walking at fixed speed.

*T* (s)	0.2	0.4	0.6	0.8
*A*_1_	2.1°	4.3°	6.5°	8.6°
*A*_2_	6.1°	6.1°	6.1°	6.1°

## Data Availability

The data used to support the findings of this study are available from the corresponding author upon request.

## References

[1] Hui-Shu M. A., Liu Y. X., Fang J. J., Luo D. W. (2019). Research on bionic foot-end trajectory planning for bionic quadruped robot.

[2] Lei J., Yu H., Wang T. (2016). Dynamic bending of bionic flexible body driven by pneumatic artificial muscles (PAMs) for spinning gait of quadruped robot. *Chinese Journal of Mechanical Engineering*.

[3] Song M. J., Ding C. J., Yu C. J. (2015). Workspace analyzing for hybrid serial-parallel mechanism of a new bionic quadruped robot. *Applied Mechanics & Materials*.

[4] He J., Gao F. (2015). Type synthesis for bionic quadruped walking robots. *Journal of Bionic Engineering*.

[5] Li M., Jiang Z., Wang P., Sun L., Ge S. S. (2014). Control of a quadruped robot with bionic springy legs in trotting gait. *Journal of Bionic Engineering*.

[6] Biswal P., Mohanty P. K. (2021). Development of quadruped walking robots: a review. *Ain Shams Engineering Journal*.

[7] Loc V.-G., Roh S.-g., Koo I. M. (2010). Sensing and gait planning of quadruped walking and climbing robot for traversing in complex environment. *Robotics and Autonomous Systems*.

[8] Hu N., Li S., Huang D., Gao F. (2014). Crawling gait planning for a quadruped robot with high payload walking on irregular terrain. *IFAC Proceedings*.

[9] Deng H., Xin G., Zhong G., Mistry M. (2017). Gait and trajectory rolling planning and control of hexapod robots for disaster rescue applications. *Robotics and Autonomous Systems*.

[10] Zhang C., Zou W., Ma L., Wang Z. (2020). Biologically inspired jumping robots: a comprehensive review. *Robotics and Autonomous Systems*.

[11] Li J., Wang J., Yang S. X., Zhou K., Tang H. (2016). Gait planning and stability control of a quadruped robot. *Computational Intelligence and Neuroscience*.

[12] Kamimura T., Aoi S., Tsuchiya K., Matsuno F. (2018). Body flexibility effects on foot loading in quadruped bounding based on a simple analytical model. *IEEE Robotics and Automation Letters*.

[13] Zhang Q., Long Z. (2017). Structure design and kinematics analysis of bionic quadruped robot. *Ordnance Industry Automation*.

[14] Winkler A. W., Farshidian F., Neunert M., Pardo D., Buchli J. Online walking motion and foothold optimization for quadruped locomotion.

[15] Focchi M., Del Prete A., Havoutis I., Featherstone R., Caldwell D. G., Semini C. (2017). High-slope terrain locomotion for torque-controlled quadruped robots. *Autonomous Robots*.

[16] Payandeh S., Majd V. J., Shoili S. M., Moghaddam M. M. Improving the stability of gait planning for quadruped robots.

[17] Sabelhaus A. P., Van Vuuren L. J., Joshi A. (2018). Design, simulation, and testing of a flexible actuated spine for quadruped robots. https://arxiv.org/abs/1804.06527.

[18] Bao-Ling H., Qing-Qiang W., Yan J., Qing-Sheng L., Chen A. Z. (2018). Trot gait planning method for improving the stability of quadruped robot. *Transactions of Beijing Institute of Technology*.

[19] Chen T., Rong X., Li Y., Ding C., Chai H., Zhou L. (2018). A compliant control method for robust trot motion of hydraulic actuated quadruped robot. *International Journal of Advanced Robotic Systems*.

[20] Zhang C., Zhang C., Dai J. S., Qi P. (2019). Stability margin of a metamorphic quadruped robot with a twisting trunk. *Journal of Mechanisms and Robotics*.

[21] Gor M. M., Pathak P. M., Samantaray A. K., Yang J. M., Kwak S. W. (2018). Fault accommodation in compliant quadruped robot through a moving appendage mechanism. *Mechanism and Machine Theory*.

[22] Gor M. M., Pathak P. M., Samantaray A. K. (2018). Development of a compliant legged quadruped robot. *Sādhanā*.

[23] Kong X. D., Ba K. X., Yu B., Li C. H., Zhu Q. X., Li W. F. (2017). The mathematical modeling and dynamic trot gait simulation on the single leg hydraulic drive system of the quadruped robot. *Applied Mechanics & Materials*.

[24] Raheem F. A., Flayyih M. K. (2017). Comparative study between classical and optimized stability margins of quadruped robot creeping gait. *American Scientific Research Journal for Engineering, Technology, and Sciences (ASRJETS)*.

[25] Yong S., Teng C., Yanzhe H., Xiaoli W. (2017). Implementation and dynamic gait planning of a quadruped bionic robot. *International Journal of Control, Automation and Systems*.

[26] Lin J., Deng G., Chen L., Jin B., Sun C., Zhang A. Bionic architecture design and robust rough-terrain locomotion for a high-payload quadrupedal robot.

[27] Lang L., Wang J., Ma H., Wei Q. Dynamic stability analysis of a trotting quadruped robot on unknown rough terrains.

[28] Li Z., Ge Q., Ye W., Yuan P. (2015). Dynamic balance optimization and control of quadruped robot systems with flexible joints. *IEEE Transactions on Systems, Man, and Cybernetics: Systems*.

[29] Zhang X., Lang L., Wang J., Ma H. The quadruped robot locomotion based on force control.

[30] Xiuli Z., Haojun Z., Xu G., Zhifeng C., Liyao Z. A biological inspired quadruped robot: structure and control.

[31] Vishal D., Manivannan P. V. (2016). Multi-body dynamics simulation and gait pattern analysis of a bio-inspired quadruped robot for unstructured terrains using adaptive stroke length. *Artificial Life & Robotics*.

